The article "Preparation of an Intelligent pH Film Based on Biodegradable Polymers for Monitoring the Food Quality and Reducing the Microbial Contaminants" was retracted in 2024. Reasons: signs of a paper mill; suspected computer-generated content; unreliable results or conclusions; concerns about the data.

# Preparation of an Intelligent pH Film Based on Biodegradable Polymers for Monitoring the Food Quality and Reducing the Microbial Contaminants

**DOI:** 10.1155/2022/7975873

**Published:** 2022-06-20

**Authors:** Kumaran Subramanian, Deivasigamani Balaraman, Kumaravel Kaliyaperumal, V. Devi Rajeswari, K. Balakrishnan, P. Ronald Ross, Elumalai Perumal, Pugazhvendan Sampath Renuga, Mani Panangal, Y. Swarnalatha, S. Velmurugan

**Affiliations:** ^1^Centre for Drug Discovery and Development, Sathyabama Institute of Science and Technology, Chennai, Tamil Nadu 600119, India; ^2^CAS in Marine Biology, Annamalai University, Cuddalore, Tamil Nadu, India; ^3^National Navel Orange Engineering Research Centre, School of Life Sciences, Gannan Normal University, Ganzhou, Jiangxi, China; ^4^Department of Biomedical Sciences, School of Biosciences and Technology VIT, Vellore, Tamil Nadu, India; ^5^Department of Zoology, Government Arts College (A), Karur, Tamil Nadu, India; ^6^Department of Zoology, Annamalai University, Annamalai Nagar, Cuddalore, Tamil Nadu, 608002, India; ^7^Departments of Pharmacology, Saveetha Dental College and Hospital, Chennai, Tamil Nadu, India; ^8^Department of Zoology, Annamalai University, Annamalai Nagar, Cuddalore, Tamilnadu 608002, India; ^9^Department of Biotechnology, Annai College of Arts & Science, Kumbakonam, Tamil Nadu, India; ^10^Department of Biotechnology, Sathyabama Institute of Science and Technology, Chennai, Tamil Nadu 600119, India; ^11^Department of Biology, School of Natural Science, Madawalabu University, Oromiya Region, Ethiopia

## Abstract

Hydrogel refers to a three-dimensional cross-linked polymeric network made of synthetic or natural polymers that can hold water in its porous structure. The inclusion of hydrophilic groups in the polymer chains, such as amino, carboxyl, and hydroxyl groups, contributes to the hydrogel's water-holding ability. At physiological temperature and pH, these polymeric materials do not dissolve in water, but they do swell significantly in aqueous media. Hydrogel can be manufactured out of almost any water-soluble polymer, and it comes in a variety of chemical compositions and bulk physical properties. Hydrogel can also be made in a variety of ways. Hydrogel comes in a variety of physical shapes, including slabs, microparticles, nanoparticles, coatings, and films. Due to its ease of manufacture and self-application in clinical and fundamental applications, hydrogel has been widely exploited as a drug carrier. Contact lenses, artificial corneas, wound dressing, suture coating, catheters, and electrode sensors are some of the biomedical applications of hydrogels. The pigment color changes were observed from colorless to pale pink followed by dark reddish-pink. Anthocyanin was produced in large quantities and tested using a UV-visible spectrophotometer. At 450–550 nm, the largest peak (absorbance) was detected, indicating the presence of anthocyanin. The FTIR analysis of this study shows the different stretches of bonds at different peaks: 2918.309 (-C-H alkane stretch), 2812.12 (-C-H aldehyde weak intensity), 192320.37/cm (C-O bend), 21915.50, 2029.08/cm (-C=C arene group), 1906.94/cm (=C-H aromatics), 1797.78/cm (=C-H), 1707.94 (-C=O ketene), 1579.70, 1382.96 (C-H alkane strong bend), 889.18/cm (C-H aromatics plane bend), and 412.77/cm (-C-CI strong bond). The spectra of the PVA/chitosan film depict the peak's formation: 1571.88, 1529.55, 1500.62/cm (C-H alkene strong bend), 1492.90, 1483.26, 1467.83/cm (C-H alkene strong bond), 670.48, 443.63, 412.77/cm (-O-H carboxylic acids with great intensity), 1708.93 (-C=O ketone), and 1656.0/cm (alkenyl C=C stretch strong bond).

The article "Preparation of an Intelligent pH Film Based on Biodegradable Polymers for Monitoring the Food Quality and Reducing the Microbial Contaminants" was retracted in 2024. Reasons: signs of a paper mill; suspected computer-generated content; unreliable results or conclusions; concerns about the data.

## 1. Introduction

### 1.1. Hydrogel

Hydrogels are defined as hydrophilic, three-dimensional polymer crisscrossing alongside a correlated absorption range to 10 g/g [1]. Hydrogel has broad demand in different branches such as agriculture [2, 3], drug discovery, and water [4]. Wichterle and Lim were the first to write on the use of hydrogels in 1960 [5, 6]. Hydrogel may be a three-dimensional polymeric structure that swells when uncovered to water and incorporates covalent bonds shaped by the response of one or more monomers, connection bonds such as van der Waals interactions, and hydrogen bonds between chains. Hydrogels may take the frame of unbending molded forms (soft contact focal points), squeezed powder networks (pills or tablets for verbal ingestion), small scale particles (as bioadhesive carriers or wound treatment), coatings (on inserts or catheters), films or sheets, and typified solids and fluids [7].

Chitosan (CS) could be a characteristic polymer inferred from chitin and is copious in crab and shrimp shells [7]. The Chitosan is polycatioinic in nature, chelating properties too film-forming based on amino and hydroxyl group in the chitosan. It shows diverse natural exercises such as antimicrobial action and biodegradability [7]. To assist in preparing polymer movies, chitosan is frequently mixed with other polymers with more flexible chains, such as poly(vinyl alcohol) (PVA) [8].

PVA is an emulsifiable nontoxic manufactured polymer of versatility and tall ductile quality and flexibility, as well as low gas permeability, such as O_2_ and CO_2_. At extraordinary temperatures, PVA can have gentle water [9]. Due to its fabulous film-forming properties, PVA has been broadly utilized in the application of lean movies, such as nourishment bundling and therapeutic application. Anthocyanins are water-soluble shades found in an assortment of plants, including ruddy cabbage, blueberries, eggplants, and blooms. Depending on the pH values, they may utilize it as a color pointer. It is gotten from ruddy cabbage in specific and can extend from ruddy to purple and to blue at different pH values [10, 11]. It makes it less demanding to distinguish the nourishment quality in terms of pH. To extend the mechanical quality of cast film cross-linking substances such as sodium tripolyphosphate (STPP), glyoxal and glutaraldehyde must be included in the handling of lean polymer films.

The article "Preparation of an Intelligent pH Film Based on Biodegradable Polymers for Monitoring the Food Quality and Reducing the Microbial Contaminants" was retracted in 2024. Reasons: signs of a paper mill; suspected computer-generated content; unreliable results or conclusions; concerns about the data.

### 1.2. Polymer-Based pH Sensitivity

pH-sensitive polymers are polyelectrolytes with frail acidic or fundamental bunches in their structure that acknowledge or discharge protons in reaction to changes in pH. These polyelectrolyte acidic or fundamental bunches can be ionized in the same way as acidic or essential bunches of monoacids or monobasic acids, and, be that as it may, total ionization of these structures is more troublesome due to their bigger measure to the electrostatic impacts of other ionized bunches adjacent. In reaction to the pH of the environment, these either discharge protons or acknowledge free protons. The anionic pH-sensitive polymers are shaped on PAA or by their subordinates. These frameworks as a rule deliver anionically charged moieties at pH levels over their pKa, which can draw in emphatically charged therapeutic agents [12].

Polymers that react to pH can be straight, branched, or organized. Depending on their frameworks, they can have distinctive reactions to arrangement conditions and diverse self-assembly behaviors. The pH adjust to dendrimer-like structures of the hydrogel dsweeling. Surface adjusted with polymers permits for the creation of ionic surface and thin/thick layers as a result of pH changes. pH adjustments cause changes in polymers of different models [13]. The pH based polymeric property are useful in life science and especially in chemical industries with conceivable applications in overseen sedate conveyance, individual care, mechanical coatings, oil investigation, and water remediation, among others [14].

A few well-known polymerization strategies can be utilized to form pH-sensitive polymers. Depending on the shape of polymerization, useful bunches can be gotten to be anticipated from responding. The concealing is regularly evacuated to restore polymerization to reestablish pH-sensitive usefulness. Since the atomic weight conveyance, living polymerization is commonly utilized to make pH-sensitive polymers. A few illustrations incorporate GTP (bunch exchange polymerization), ATRP (molecule exchange radical polymerization), and reversible addition-fragmentation chain exchange (pontoon). Unite polymers, which have a spine with branches, are a common frame of the union. The department structure can be altered to attain different properties [15, 16].

The article "Preparation of an Intelligent pH Film Based on Biodegradable Polymers for Monitoring the Food Quality and Reducing the Microbial Contaminants" was retracted in 2024. Reasons: signs of a paper mill; suspected computer-generated content; unreliable results or conclusions; concerns about the data.

### 1.3. Food Packing

Nourishment bundling is one of the foremost imperative perspectives of a product from the consumer's perspective as well as one important position of the foremost vital in present-day commercial exchange [17, 18] since it guarantees nourishment quality and assurance, helps in transportation, permits secure capacity, maintains a strategic distance from item hurt and misfortune, decrease financial misfortunes, and helps in item showcasing and in a roundabout way protect consumer's well-being [13]. Conventional and common food packaging, which is made of petroleum subordinates, may be a safe gadget. It acts as an obstruction against microbial/physicochemical harm, as well as natural conditions and outside jolts, amplifying the rack life of the nourishment item [19].

Biopolymers such as proteins, polysaccharides, and their subordinates are characteristic polymers that debase within the environment as a result of common physical, chemical, and natural forms, particularly microorganism digestion systems [20, 21]. It may be isolated by an assortment of characteristic assets. Plant-based polysaccharides such as chitosan, starch, cellulose, alginate, agar, carrageenan, pectin, and different gums are commonly utilized [21]. Whereas one of the capacities of food packing is to guarantee nourishment quality and security, advanced bundling too must inform the client about nourishment quality and supportability for utilization. A few shrewd bundling frameworks based on colorimetric pointers will give shoppers real-time quality checking for nourishment things through quality sensors/indicators which are highly needed for the current situation [22].

These characteristic colorants implanted within the biopolymeric film framework show up to alter color as the physiological condition of the nourishment alters amid deterioration, educating the client of the bundled food's consistency and appropriateness for utilization in this manner. Plastic containers and tanned food items are easily contaminated by the polyethylene terephthalate constituents and tanned ores. Wrapped foods with aluminum foils are highly prone to aluminum toxicity in infants.

### 1.4. Plant Pigment

Since plant colors are displayed in each life form on the planet and plants are the essential makers, pigment creates the colors that we see in each arrangement of our lives. They can be useful in natural products, vegetables, and blooms and in skin, eyes, and other creature structures, as well as microscopic organisms and organisms. Common and manufactured shades are utilized in drugs, nourishments, dresses, furniture, beauty care products, and others [24]. Shades are chemical compounds that assimilate light within the wavelength run of the unmistakable locale. A molecule-specific structure (chromophore) is capable of delivering color. The vitality is captured by this structure, an electron is energized from an external orbital to the next orbital, the nonabsorbed vitality is reflected and or refracted to be captured by the eye, and the created neural motivations are transmitted to the brain, where they can be seen as a color [25].

The article "Preparation of an Intelligent pH Film Based on Biodegradable Polymers for Monitoring the Food Quality and Reducing the Microbial Contaminants" was retracted in 2024. Reasons: signs of a paper mill; suspected computer-generated content; unreliable results or conclusions; concerns about the data.

Colors can be classified by their root as characteristic, engineered, or inorganic. Characteristic shades are delivered by living life forms such as plants, creatures, parasites, and microorganisms. Manufactured colors are gotten from research facilities. Characteristic and manufactured colors are natural compounds. Characteristic shades such as anthocyanins can be included in biodegradable starch movies to supply the required utilitarian properties of a pH marker. Anthocyanins are auxiliary metabolites broadly conveyed in natural products and vegetables (e.g., ruddy cabbage, sweet potato, bean husk, and grapes), making them a promising source of common marker that secured a wide color range as a work of pH [26].

### 1.5. Red Cabbage Pigment

The ruddy cabbage (*Brassica oleracea*) is such a cabbage, which is recognized by its shading. The leaf of ruddy cabbage is more to some degree blue-purple versus ruddy tone. Ruddy cabbage is as of now created and traded generally as a colorant within the nourishment commerce. Anthocynains can provide the phynlpropanoid pathway with the flavonoid class [27]. Ruddy cabbage may be a wealthy origin of anthocyanins, which can be utilized for common tinge. Its tone is pH subordinate [28]. The ruddy cabbage contains 24 sorts of anthocyanins of sweet-smelling and aliphatic corrosive.

The anthocyanins have physiological capacities, like antihypertensive, cancer prevention agent limit, hepatoprotection, and antihyperglycemic impacts [29]. The prevalent anthocyanin of red cabbage is developed from cyanidin-3-Di glucoside-5-glucoside, which could be nonacylated, monoacylated, or diacylated with caffeic, p-coumaric, sialic, and ferulic acids [30]. Anthocyanins are the biggest gathering of water-solvent colorants and are liable for blue, purple, and red tones of many blossoms and leafy plant food. In this way, red cabbage could be utilized as a characteristic colorant in food enterprises [31] and as a pH marker [32].

The article "Preparation of an Intelligent pH Film Based on Biodegradable Polymers for Monitoring the Food Quality and Reducing the Microbial Contaminants" was retracted in 2024. Reasons: signs of a paper mill; suspected computer-generated content; unreliable results or conclusions; concerns about the data.

Red cabbage is of high benefit as it is plentiful in minerals, nutrients, oligosaccharides, and various bioactive substances such as anthocyanins, flavonols, and glucosinolates [33], having a positive effect on human well-being aside from various nourishing advantages. Red cabbage is likewise esteemed for its taste and for being a source of serious red shading, which expands the tasteful estimation of the food. For these reasons, red cabbage is a widely and habitually burned-through vegetable as a new cut serving of mixed greens. Likewise, red cabbage is portrayed by a high period of usability; along these lines, it very well may be effortlessly put away and accessible in a new structure lasting through the year.

### 1.6. Pigment, Gel, and Film

Red cabbage (*Brassica oleracea* L.) is a consumable source with a high substance and high potential yield per unit territory of anthocyanins [34]. Red cabbage anthocyanin removal is known to have impressive measures of mono- or diacylated cyanidin anthocyanins [35]; type and acylation of anthocyanins are two significant components that decide their shading attributes at certain pH values [36]. Due to its anthocyanin organizations, red cabbage anthocyanin concentrates can display a wide range of shading going from orange through red to purple and blue because of the pH of the environment. Acylation of anthocyanins likewise impacts their cancer prevention agent properties and strength in the food. Anthocyanins are the biggest gathering of water-solvent colorants and are liable for the blue, purple, and red tones of many blossom plant products of the soil. Red cabbage could be utilized as a characteristic colorant in food enterprises [37] and as a pH pointer.

Three-dimensional organizations of hydrophilic polymers in hydrogels stood out towards the fuse of a higher measure of medications for their application in lethargic maintained and controlled medication conveyance because of the arrangement of covalent bonds ionic communication, hydrogel holding, and hydrophobic connections [38]. Chitosan (CS) is a characteristic polymer gotten from chitin and discovered richly in the shells of crabs and shrimps [7]. Chitosan is not generally best in polymer handling for film creation attributable to its mediocre mechanical properties like lower elasticity, less lengthening-at-break, and young's modulus. Polyvinyl alcohol (PVA) is a water-dissolvable biodegradable engineered polymer with huge pliable strength, and the composites mixed with PVA and chitosan are known to have improved steadiness, biocompatibility, and mechanical strength, compared with those of unadulterated PVA and unadulterated CS polymers [8].

The article "Preparation of an Intelligent pH Film Based on Biodegradable Polymers for Monitoring the Food Quality and Reducing the Microbial Contaminants" was retracted in 2024. Reasons: signs of a paper mill; suspected computer-generated content; unreliable results or conclusions; concerns about the data.

The hot condense removal routinely requires the commitment of tall vitality, for example, mechanical vitality as greatly tall sheer weight as well as atomic control, to guarantee the arranged polymer within the mollified state. In that capacity, this method is not suitable for planning a polymer with warm and shears-sensitive particles. Alternately, dissolvable anticipating is the predominant procedure for collecting movies containing temperature-delicate fixings, for example, anthocyanin, since the temperature required to disappear the dissolvable is frequently lower than the cycle temperature of the hot melt ejection [39, 40].

### 1.7. Food Packing-pH Film

A long time later, there has been an increment in open concern almost the transfer of conventional manufactured plastics, especially when the whole time of the plastic debasement is exceptionally long. Numerous considerations looked into biodegradable movies, such as eatable films and coating made from eatable materials, with the trust of moving forward the quality of food products and expanding their rack [41]. Chitosan could be a natural cationic polysaccharide and a diacylated chitin subordinate inferred fundamentally from shellfish handling squander. Chitosan has antimicrobial properties, which suggests it can halt organisms, yeast, and microbes from developing. Chitosan film has been found to have tall mechanical quality, adaptability, biodegradability, and antibacterial properties [42].

The nourishment industry has contributed to keen bundling in the rack in reaction to a client's request for fresher things with a longer rack life. The bundling savvy with pH markers was made with the point of empowering a considered relationship between nourishment and bundling in arrange to make strides in quality characteristics. Because it is caught on that nourishment disintegration is linked to pH changes within the item, buyers can identify these changes within the nourishment by basically altering the color of the bundling [43].

Since plastic is commonly utilized in numerous applications, dietary packing, the improvement of pH marker bundling can come from either fossil or renewable sources. Plastic, on the other hand, includes an inconvenient impact on the climate since it contaminates the environment and is not biodegradable plastic utilizing starch, alginate, and normal filaments, for example, which can be utilized as food coatings due to their degradable properties and preservation capacity, maybe a progressive arrangement to this issue pointed at natural conservation and halfway substitution of conventional polymers inferred from unrefined oil [44].

The article "Preparation of an Intelligent pH Film Based on Biodegradable Polymers for Monitoring the Food Quality and Reducing the Microbial Contaminants" was retracted in 2024. Reasons: signs of a paper mill; suspected computer-generated content; unreliable results or conclusions; concerns about the data.

The present research is to create a food packing film made entirely of sustainable and biodegradable materials. As a result, chitosan (CS) was chosen as a partial replacement for poly(vinyl alcohol) (PVA) in the packing film. Furthermore, anthocyanin (ATH), a food colorant widely used [45] and extracted from red cabbage in this analysis, is added to the cast film for acclimatization.

## 2. Materials and Methods

### 2.1. Preparation of Cabbage Extract

Red cabbage (*Brassica Oleracea* L.) was obtained from a local store in Chennai, Tamil Nadu. Using water and ethanol as solvents, extraction from red cabbage was made. 25 g red cabbage, 50 ml water, and 50 ml ethanol were chopped and combined in a chopper (96 percent), and 1% of HCL was added. The extract was then given 50 mL of additional solvent and stirred for half an hour at 300 rpm. Finally, coarse particles were removed with a strainer before filtering with filter paper (Whatman no. 1). Depending on whether the solvent used to extract anthocyanins was water (w) and ethanol (e), these extracts were given the names Aw and Ae. The extracts were then centrifuged at 6000 rpm for 15 mins.

### 2.2. Characterization of Red Cabbage Extract

#### 2.2.1. Total Anthocyanins Concentration

A 200 *µ*l aliquot of anthocyanin extract was combined with 7 ml of pH 1.0 buffer (0.025 M potassium chloride changed with hydrochloric acid) and 7 ml of pH 4.5 buffer (acetate of sodium 0.4, adjusted with w/w with acetic acid). The difference in absorbance between the two buffers at 530 nm (maximum absorption wavelength) is proportional to the anthocyanin material [46]. Using distilled water as a blank, measurements were made on a UV-Vis plate reader. Corrections were made using the absorbance at 700 nm to account for the presence of damaged compounds or interfering substances. Since red cabbage anthocyanins are derived from cyanidin glucoside, concentrations were expressed as mg cyanidin-3-glucoside per 100 ml extract and calculated using the following equation:

(1) $$\begin{array}{c} \text{Anthocyanin concentration}=\frac{\Delta A\cdot MW\text{ average}\cdot FD\cdot 1000}{\varepsilon \cdot \text{L}},\\ 112\Delta A=\left(A530-A700\right)pH:1,0-\left(A530-A700\right)pH:4.5, \end{array}$$

where *A* is the distinction between the absorbance move at 530 and 700 nm in buffers with pH 1 and 4.5; *MW* normal is the atomic mass of cyanidin-3-glucoside (449.2 g/Mol); FD is the cyanindin-3-glucoside molar absorbance (26,900) *L* is the optical way (cm); 1000 is the change calculate of grams to milliequivalent taken three times.

### 2.3. Preparation of Film

The casting technique was used to prepare the film. Until combining the two solutions, the PVA and chitosan solutions were prepared separately. The chitosan solution was made using a literature review [47]. 1% of hydrogel was prepared as 2 g of chitosan powder was dissolved in 2 mL of the acetic acid solution and 1 percent sodium tripolyphosphate in 100 mL distilled water, and the mixture was mixed under magnetic stirring at room temperature. To achieve maximum dispersion of the chitosan, the solution was stirred for 24 hours at 650 rpm until the entire chitosan flake disappeared. 2 g of PVA and 100 mL distilled water were mixed with a magnetic stirrer at 100°C for 30 minutes at 650 rpm until the PVA solution homogenized and gelatinized. Following that, the prepared PVA and chitosan solutions were combined with 25 mL of red cabbage extract. The blended solution was stirred at room temperature for 24 hours to ensure that it was thoroughly mixed. Afterward, 20 mL of the fibrogenic solution was spread on a plated dish and dried for 48 hours at 40 degrees Celsius in a dryer with forced air convection. Before the other checks, the dried film was conditioned in a desiccator.

The article "Preparation of an Intelligent pH Film Based on Biodegradable Polymers for Monitoring the Food Quality and Reducing the Microbial Contaminants" was retracted in 2024. Reasons: signs of a paper mill; suspected computer-generated content; unreliable results or conclusions; concerns about the data.

### 2.4. Confirmatory Test of Anthocyanin

By taking 1 mL of sulfuric acid in a test tube that contains 2 mL of red cabbage extract and keeping this for minutes, it shows the color changes from rose to orange color. This indicates the presence of anthocyanin.

### 2.5. Sodium Hydroxide Test

Take 1 mL of 1 N NaOH in a test tube, with the addition of 2 mL of red cabbage extract. This shows the color changes from rose to a bluish-green color.

### 2.6. Characterization of Chitosan

#### 2.6.1. Fourier Transform Infrared (FTIR) Spectroscopy

Fourier Transform Infrared (FTIR) study was utilized to degree the atomic cohesion between poly (vinyl alcohol) and chitosan. The atomic intuition of all the tests, counting manufactured polymer powdered and hydrogel movies arranged employing an arrangement casting strategy, was measured utilizing Fourier change infrared (FTIR) spectroscopy. FTIR spectra of all the tests were obtained utilizing an Alpha *E* ATR-FTIR, Bruckner, Germany, with wave numbers extending from 400 to 4000 cm^−1^.

#### 2.6.2. Scanning Electron Microscopy

The surface morphology of the prepared hydrogel membrane was studied using scanning electron microscopy (SEM). The established hydrogel was examined using an FEI QUANTA 450 Scanning Electron Microscope at 4.00 *k* x magnification. The hydrogel layer was freeze-dried for 24 hours before SEM research, and then the surface was coated with gold (Kaushal Kumar Mahato et al., 2019).

#### 2.6.3. Particle Size Analysis

Molecule estimate examination could be a strategy for deciding the molecule estimate dispersion in a fabric. Strong materials, suspensions, emulsions, and indeed pressurized canned products can take all advantage from molecule size analysis. Molecule measures can be measured by employing an assortment of strategies.

The article "Preparation of an Intelligent pH Film Based on Biodegradable Polymers for Monitoring the Food Quality and Reducing the Microbial Contaminants" was retracted in 2024. Reasons: signs of a paper mill; suspected computer-generated content; unreliable results or conclusions; concerns about the data.

Particle size analyzers (PSA) are machines that quantify particle size using a variety of technologies, including high-resolution image processing, Brownian motion analysis, particle gravitational settling, and light scattering (Rayleigh and Mie scattering).

## 3. Results

### 3.1. Confirmatory Test of Anthocyanin

The existence of anthocyanin was confirmed chemically due to the formation of the reddish-orange color of the solution upon the addition of H_2_SO_4_ (Figure 1). The dark-bluish solution was also observed upon the addition of 1 N NaOH, which quickly changed (Figure 2). Since anthocyanin types are pH-based, confirmatory tests for anthocyanins use acidic and basic solutions. When anthocyanins react with acids and bases, they undergo molecular transformations. In an acidic medium, the flavylium ions are the most common type which produce a red color.

### 3.2. Synthesis and Chemical Characteristics of pH Indicative Film

Anthocyanin (ATH) was extracted successfully from red cabbage.  Figure 3 depicts the color shift in buffer solution from pH 1 to pH 13 with an ATH concentration of 86.67 mg/L. One benefit of using anthocyanin as a pH predictor is the visible shift in color as they come into contact with various pH values. In acidic solutions, they are red or pink, while in alkaline solutions, they are blue or green. ATH was developed as a pH indicator and was used to create pH indicator films made of PVA, CS, and STPP (Figure 4). The color change due to pH changes from acidic to basic is due to ionic changes in the sample.

### 3.3. Fourier Transform Infrared (FTIR) Spectroscopy

The result of the FTIR analysis of this study (Figure 5) shows different stretches of bonds shown at different peaks: 2918.30 (-C-H alkane stretch), 2812.12 (-C-H aldehyde weak intensity), 2320.37/cm (C-O bend), 2191.50, 2029.08/cm (-C=C arene group), 1906.94/cm (=C-H aromatics), 1797.78/cm (=C-H), 1707.94 (-C=O ketone), 1579.70, 1382.96 (C-H alkane strong bend), 889.18/cm (C-H aromatics out of the plane bend), and 412.77/cm (-C-CI strong bond).

The results of the FTIR analysis of this study (Figure 6) show different stretches of bond shown at different peaks: 2360.87/cm (-O-H carboxylic acids with strong intensity), 1708.93 (-C=O ketone), 1656.0/cm (alkenyl C=C stretch (alkene) olefinic), 1571.88, 1529.55, 1500.62/cm (C-H alkene strong bend), 1492.90, 1483.26, 1467.83 (C-H alkene strong bend), 670.48, 443.63, and 412.77/cm (-C-CI strong bond).

The article "Preparation of an Intelligent pH Film Based on Biodegradable Polymers for Monitoring the Food Quality and Reducing the Microbial Contaminants" was retracted in 2024. Reasons: signs of a paper mill; suspected computer-generated content; unreliable results or conclusions; concerns about the data.

### 3.4. SEM Analysis

The SEM pictures (Figures 7 and 8) for chitosan film before and after anthocyanin pigments adsorption show that the film surface was coated, and the film roughness was reduced. This is due to the deposition of anthocyanin molecules on the surface of the material.

The goal of *Brassica oleracea* in the present research was to find out how important the product's life cycle is. The red cabbage was taken out of the ground and identified. The findings are noteworthy in a novel way and would be a helpful product for society.

By adding H_2_SO_4_, a confirmatory test for anthocyanin derived from red cabbage results in the production of a reddish-orange color. The addition of 1 N NaOH results in a dark-bluish color. Variation is to be expected. When color changes were seen, they varied slightly based on the type of anthocyanin. Anthocyanin was extracted using acidic ethanol, and vivid red was detected. When H_2_SO_4_ is added, the solution turns reddish-orange, and when 1 N NaOH is added, the solution turns bluish-green and shortly turns yellowish-brown. FTIR analysis is analyzed to determine the interactions between PVA, chitosan, and red cabbage extract by observing the changes in the peak positions or wave numbers of the functional groups that exist in the spectrum.

The spectra of a PVA/Chitosan anthocyanin film are shown in (Figure 9). The absorption peaks formed by the functional groups contained in the composite film can be categorized based on the raw materials component. The peaks are 2918.309 (-C-H alkane stretch), 2812.12 (-C-H aldehyde weak intensity), 192320.37/cm (C-O bend), 21915.50, 2029.08/cm (-C=C arene group), 1906.94/cm (=C-H aromatics), 1797.78/cm (=C-H), 1707.94 (-C=O ketene), 1579.70, 1382.96 (C-H alkane strong bend), 889.18/cm (C-H aromatics plane bend), and 412.77/cm (-C-CI strong bond). The spectra of PVA/Chitosan film are shown in (Figure 10). It depicts the peak's formation: 1571.88, 1529.55, 1500.62/cm (C-H alkene strong bend), 1492.90, 1483.26, 1467.83/cm (C-H alkene strong bond), 670.48, 443.63, 412.77/cm (-O-H carboxylic acids with great intensity), 1708.93 (-C=O ketone), and 1656.0/cm (alkenyl C=C stretch strong bond). In research by Suzihaque M.U.H et al. 2019, the absorption peaks at 3285.07 cm^−1^ indicate modest changes in peak development (O-H stretching and N-H stretching). The composite film was to blame for the N-H stretching. The alkane group is represented by 2933.77 cm^−1^ (C-H_2_ stretching), the amide band is represented by 1645.92 cm^−1^ (C=O stretching), the CH_2_ group is represented by 1410.82 cm^−1^ (C-H bending variations), the ester group is represented by 1151.30 cm^−1^ (C-O stretching), the ester group is represented by 1025.86 cm^−1^ (C-O-C stretching).

The article "Preparation of an Intelligent pH Film Based on Biodegradable Polymers for Monitoring the Food Quality and Reducing the Microbial Contaminants" was retracted in 2024. Reasons: signs of a paper mill; suspected computer-generated content; unreliable results or conclusions; concerns about the data.

When placed at different pH levels, a good indicator film can show a variety of striking color changes. The most significant part of manufacturing the indication film is this function. The indicator film must be able to produce color changes that are visible to the naked eye. The primary goal of using film indicators in food packaging is to monitor food quality by measuring changes in pH without having to open the package or replace the product.

The chitosan-PVA film has limitations in the application for dry food kinds of stuff, despite its capacity to signal food spoilage. The fil must come into direct touch with the food surface and contain enough water to soak into the polymer film. Furthermore, this film should be used on a product that is maintained in a chiller or freezer to prevent anthocyanin extract from being damaged by high temperatures.

## 4. Discussion

Hydrogel things set up a gathering of polymeric materials, the hydrophilic plan of which makes them prepared for holding a parcel of water in their three-dimensional systems [48]. The broad work of these things in different present-day and biological spaces of utilization is seen as of prime centrality. Composing concerning this matter was discovered to amplify, especially within the consistent spaces of investigation. The basic target of this paper is to review the composition concerning the course of action of hydrogels on different bases, the physical and compound qualities of these things, and the specialized achievability of their utilization. It moreover expands developments grasped for hydrogel creation at the side degree and arranges proposals, square traces, and progressed states of the status interaction. A progressed classification of progressing ages of hydrogel materials was also presented in certain subtleties.

Haghighia [49] clarified that the later sharp rise in the introduction to natural concerns emerging from plastic bundling has started intrigued in more naturally neighborly bundling materials. This most recent slant energizes the commercialization of data through the utilization of chitosan-based films.

Because of its unordinary natural and useful properties, chitosan has been broadly inquired about and utilized; in any case, inalienable imperfections such as a moo mechanical properties and tall helplessness to stickiness confine its mechanical applications, which incorporate nourishment bundling. Chitosan and poly(vinyl alcohol) (PVA) were utilized to make a semi-interpenetrating polymeric organize that was cross-linked with glutaraldehyde. The chitosan had an atomic weight of 612 kDa and a degree of deacetylation of 72 percent, individually [50]. The chemical bonds shaped by cross-linking response were examined, as well as their change in completely different pH media. The mechanical properties of the hydrogel and the gelatin property of the chitosan-PVA gel arrangement were explored. The arrangement of Schiff's base (C=N) and -NH_3_^+^ was recommended by the FTIR spectra of the hydrogel sometime recently and after swelling at pH 3 and pH 7. They too illustrated the pH-induced change of C=N to C-N and -NH_3_^+^ to -NH_2_, as well as Schiff's base's precariousness. The chitosan is required to frame hydrogel arrangement due to Schiff's base response between the chitosan amino bunches and the glutaraldehyde bunches. The expansion of PVA improved the hydrogel's mechanical properties. PVA on the other hand shows up to filter out within the acidic medium amid longer swelling periods due to hydrolysis of the gel systems, Schiff's establishment. Alizadeh-Sani et al. [51] clarified that the unused rising in nature with secure nourishment and changing buyer viewpoints had procured advancements in packaging development. Clients are continuously asking for common nourishment colorants like carotenoids, betadine, anthocyanins, and chlorophylls rather than designed colors for nourishment applications. Appropriately, canny bundling subordinate on characteristic colorants and biopolymers has been displayed as the foremost later advancement within the nourishment bundling field. Sharp things shield nourishment from common dangers; additionally, they convey progressing messages (colorimetric, engineered, or electrical) to customers for changes within the bundling climate and nourishment quality.

The article "Preparation of an Intelligent pH Film Based on Biodegradable Polymers for Monitoring the Food Quality and Reducing the Microbial Contaminants" was retracted in 2024. Reasons: signs of a paper mill; suspected computer-generated content; unreliable results or conclusions; concerns about the data.

Pigments are available in all living matter and give appealing tones and assume fundamental parts in the development of organic entities. People, like most creatures, interact with their environmental factors through shading, and things can or cannot be adequate depending on their shading qualities [52]. This audit presents the essential data about colors zeroing in consideration on the common ones; it underscores the chief plant shades: carotenoids, anthocyanins, and betalains. Exceptional contemplations are given to their striking attributes, to their striking attributes, to their biosynthesis, considering the biochemical and atomic science data produced in their explanation, and to the handling and soundness properties of these mixtures as food colorants.

Anthocyanins shades are fitting as standard colors for nourishment, cosmetics, and dietary improvements, since of the intrigued for superior things and their cancer avoidance specialist properties. This work implied removing the anthocyanin colors from ruddy cabbage and its segment of the course of action by adsorption movement onto chitosan movies. The anthocyanins were removed from ruddy cabbage in hot water at 90°C for 15 min. Chitosan was gotten from shrimp squander, and its movies were made by anticipating strategy (inflexibility of 25.1 ± 1.9 Mpa, extending of 10 ± 3.5%, and thickness of 103.1 ± 1.3 *µ*m). The anthocyanin adsorption tests acted in clusters, and the foremost vital assimilation constraint was around 140 mg·g^−1^. The balance trail information was changed by Henry, Langmuir, and Freundlich models, and all models showed a decent fitting (*R*2 ≥ 0.96 and ARE ≤6.5%). The thermodynamic boundaries addressed endothermic and actual adsorption. The dynamic conduct was assessed by exact models, being the pseudofirst request model that showed the best fitting (*R*2 ≥ 0.97 and is ≤ 8.5%). This work introduced reasonable data about the anthocyanin molecule immobilization onto chitosan films, and these outcomes could be critical to the utilization of these pigments with chitosan in various zones [53].

The article "Preparation of an Intelligent pH Film Based on Biodegradable Polymers for Monitoring the Food Quality and Reducing the Microbial Contaminants" was retracted in 2024. Reasons: signs of a paper mill; suspected computer-generated content; unreliable results or conclusions; concerns about the data.

Musso et al. [54] explain that the point of this work was to create a biodegradable protein-based film fit for sense pH changes. These protein films were set up by projecting from fluid arrangements like gelatin, glycerol, and three corrosive base markers: methyl orange (MO), nano red (NR), and bromocresol green (BCG), at pH 2.6 and 11. All consequent protein movies were homogeneous and slim and had different tones depending upon pH and the pointer utilizer. The response of these materials was evaluated by creating their contact with liquid and semisolid media and with a compartment headspace at destructive and solvent pH. In all tests, made protein movies may alter their shading within the mix of being in contact with media of different pH. The physicochemical properties of movies were moreover impacted contrastingly by the nearness of each destructive base marker.

Chitosan and starch are biodegradable polymers with solid film-forming properties and a wide run of applications within the nourishment industry, counting dynamic and savvy bundling that can track and warm clients almost nourishment conditions in genuine time. As a result, we display a pH checking framework based on chitosan, corn, starch, and ruddy cabbage extract, all of which can be gotten cheaply from renewable sources. The device was characterized using TG-DSC, FTIR, water vapor transmission rate, and light microscopy. Application tests with fish fillets were performed to verify the use of this device as a fish spoilage detection sensor. These results show that the device has strong optical and morphological properties and is extremely sensitive to pH changes. The machine visually indicated pH changes during the application test. Since the system exhibits a clear response to changes in sample pH, it could be used as a visual indicator of food storage and consumption conditions. Polysaccharides and proteins are abundant in nature and, due to their unique properties, are highly recommended for the production of environmentally friendly materials. However, due to poor mechanical and physical properties, they sometimes fail to meet basic specifications. PVA (polyvinyl alcohol) is a promising synthetic polymer with superior properties that can be blended with natural polymers to create new biomaterials with better performance [55].

The article "Preparation of an Intelligent pH Film Based on Biodegradable Polymers for Monitoring the Food Quality and Reducing the Microbial Contaminants" was retracted in 2024. Reasons: signs of a paper mill; suspected computer-generated content; unreliable results or conclusions; concerns about the data.

Intriguing bundling can emanate a flag in genuine time in reaction to any change within the starting bundling conditions and nourishment quality, in expansion to acting as a nourishment security obstruction. The colorimetric sensor in pH markers or pH sensors is ordinarily made up of two parts: a strong base and color to alter the pH level. The colors are determined from an assortment of natural products and vegetables, as well as synthetics. The pH of nourishment changes at the beginning of the corruption preparation; this move is one of the measures of product quality. Packaging with a pH pointer could be a security measure that can mean the consistency of the nourishment at the time of buying or earlier than utilization [56].

pH characteristic movies were effectively synthesized from hydrogels made by combining 1% poly(vinyl alcohol) (PVA) and 1% chitosan (CS) with anthocyanin (ATH) and sodium tripolyphosphate in this sample (STTP). To make strides in the mechanical properties of the cast movies, ATH extracted from ruddy cabbage was utilized as the pH marker, and STTP was utilized as the cross-linking specialist. The nearness of the ATH within the cast movies was confirmed by FTIR spectra. The cast film's malleable quality, elongation-at-break, and swelling records were too decided. The compositions of PVA/CS and the STPP dose connected within the hydrogels had a noteworthy effect on the properties of pH demonstrative movies. On the off chance that 35 percent of the PVA hydrogel was supplanted with CS, the malleable quality of a film cast from unadulterated PVA hydrogel seems to drop from 43.27 MPa to 29.89 Mpa. The cast films were utilized as a nourishment wrap that might be utilized to outwardly track the consistency of the enwrapped nourishment by changing color as the pH values of the enwrapped nourishment change. In hone, a consecutive move in color on the pH suggestive movies in part enwrapping the pork paunch was effectively watched, signaling the meat's deterioration [57, 58].

The article "Preparation of an Intelligent pH Film Based on Biodegradable Polymers for Monitoring the Food Quality and Reducing the Microbial Contaminants" was retracted in 2024. Reasons: signs of a paper mill; suspected computer-generated content; unreliable results or conclusions; concerns about the data.

Hydrogels made of cellulose, which contain an assortment of natural biopolymers such as cellulose, chitin, and chitosan, are hydrophilic materials that can assimilate and hold an expansive sum of water in their interstitial locales. These polymers have a wide extent of exceptional properties, counting pH, time, temperature, chemical species, and organic conditions responsiveness, as well as tall water assimilation capacity. Biopolymers hydrogels can be controlled and planned for an assortment of applications. Due to their biocompatibility, biodegradability, and wealth, analysts all over the world are centering on normally inferred hydrogels in reaction to expanding natural issues and requests [58]. The hydrogels made of cellulose are called biocompatible materials that can be used in medical devices to treat, supplement, or replace any tissue, organ, or body function. These hydrogels seem moreover to be utilized in rural exercises, as keen materials, and for an assortment of others. This audit gives an outline of later and current ponders on the physiochemical properties of cellulose-based hydrogels, as well as their applications in biomedical areas such as medicate conveyance, tissue designing and wound recuperating, healthcare and clean items, horticulture, materials, and mechanical applications as shrewd materials [59]. Red cabbage is a vegetable known for its improved bioactive constituents. It is utilized as fixing in crude servings of mixed greens [60]. It is broadly utilized in nourishment generation to move forward the stylish esteem of nourishment and to supply well-being benefits as a common colorant in drinks, candies, and gums. It has numerous well-being benefits, counting security against cancer and diabetes, as well as fortifying the resistance framework, helping in body detoxification, advancing weight misfortune, making strides skin, decreasing aggravation, and soothing clogging [61].

This minireview provides a brief overview of the reasons for red cabbage's popularity in agriculture, as well as why we should encourage growers to concentrate on the production technologies associated with the cultivation process. The crop not only is tasty but also has a lot of advantages. The point of this inquiry is to make strides in the characteristics and pertinence of these markers. This survey paper incorporates the ponders on shades, polymers, nourishment, and bundling arrangement, as well as an outline of the materials/technologies utilized within the generation and the perspectives/challenges that this modern innovation brings.

The article "Preparation of an Intelligent pH Film Based on Biodegradable Polymers for Monitoring the Food Quality and Reducing the Microbial Contaminants" was retracted in 2024. Reasons: signs of a paper mill; suspected computer-generated content; unreliable results or conclusions; concerns about the data.

## 5. Conclusion

The pH characteristic sensors comprised of PVA/CS/ATH have been effectively cast from hydrogels by mixing 1 percent PVA arrangement and 1 percent CS arrangement in different volume proportions, doped with ATH as a pointer, and blended with STPP as a cross-linker. These films have palatable mechanical properties and show fast colors that alter pH buffers. Ruddy cabbage extract had more potential as a pH pointer bundle. Red cabbage extracts with gel polymer make a good food quality indicator. This will offer a clear picture of the system's real-world potential as a portion of savvy nourishment bundling.

## Figures and Tables

**Figure 1:** Sulfuric acid (H_2_SO_4_) test.

**Figure 2:** Sodium Hydroxide test of anthocyanin.

**Figure 3:** Color change of anthocyanin from pH 1 (left) to pH 13 (right).

**Figure 4:** Preparation of pH film.

**Figure 5:** FTIR analysis spectrum of PVA/CS/ATH.

**Figure 6:** FTIR analysis spectrum of PVA/CS.

**Figure 7:** Circular dichroism of PVA/CS.

**Figure 8:** The spectra of PVA/Chitosan.

**Figure 9:** SEM image of Sample 1.

**Figure 10:** SEM image of Sample 2.

## Data Availability

The data used to support the findings of this study are included in the paper.
